# N-Acetylcysteine (NAC) Inhibits Synthesis of IL-18 in Macrophage by Suppressing NLRP3 Expression to Reduce the Production of IFN-*γ* from NK Cells

This article has been retracted.

**DOI:** 10.1155/2021/7596343

**Published:** 2021-12-03

**Authors:** Xiaopeng Liu, Xufeng Lu, Zhixiong Hu

**Affiliations:** Department of Respiratory Medicine, Jinshan Hospital, Fudan University, Shanghai 201508, China

## Abstract

**Background:**

N-Acetylcysteine (NAC) had exerted antioxidation and anti-inflammation effects on chronic obstructive pulmonary disease (COPD) patients. However, its effect in regulating interleukin- (IL-) 18 was not fully understood. This study was designed to evaluate the specific mechanism of NAC regulating IL-18.

**Materials and Methods:**

A total of 112 COPD patients and 103 health individuals were recruited in the study. Cytokine level in patients' serum was measured by enzyme-linked immunosorbent assay (ELISA). A COPD mouse model was established by administration of lipopolysaccharide (LPS) and cigarette smoke. The expression of cytokines was measured by ELISA and flow cytometry. Inflammasome-related protein was measured by Western blot.

**Result:**

NAC could effectively improve the immune status of COPD patients as well as the COPD mouse model by downregulating proinflammation and inflammation cytokines including IL-1*β*, interferon- (IFN-) *γ*, tumor necrosis factor- (TNF-) *α*, and IL-18. It also had the capability to suppress synthesis of IL-18 in macrophage to inhibit the secretion of IFN-*γ* from natural killer (NK) cells through influencing the inflammasome-related protein in macrophages.

**Conclusion:**

NAC could effectively inhibit the production of IL-18 by suppressing NLRP3 expression in macrophages to reduce the production of IFN-*γ* in NK cells.

## 1. Introduction

Chronic obstructive pulmonary disease (COPD) is one of common chronic respiratory diseases, which is comprised of several classical clinical feature such as chronic airflow obstruction, usually progressive and almost irreversible, chronic bronchitis caused by inhalation, and small airway damage. The prevalence of this fatal disease is increasing dramatically worldwide, which is expected to be the third-leading cause of death, placing a great burden on world's disease economy [1, 2].

N-Acetylcysteine (NAC) is a mucolytic and antioxidant drug that may also influence several inflammatory pathways. It provides the sulfhydryl groups and acts both as a precursor of reduced glutathione and as a direct reactive oxygen species (ROS) scavenger, hence regulating the redox status in the cells. Oral NAC had proven its effect on reducing the oxidation and inflammation in the lung and peripheral blood and exhaling breath condensate, as well as reducing the rate of COPD deterioration [3–5].

In recent years, more and more studies tended to clarify the inflammation-related mechanisms in COPD, especially the complex regulatory mechanism of cytokines. Cytokines play a significant role in the formation of inflammation and pathophysiological mechanisms of airway obstruction in both asthma and COPD. TNF-*α* is one of the classic proinflammatory molecules involved in the development of COPD and bronchial asthma (BA) [3, 6]. At the present stage, experimental data and results of clinical studies on the possible involvement of phlogogenic molecules such as IL-17 and IL-18 in the genesis of airway obstructive diseases have appeared [6–8]. Interleukin-17 (previously known as IL-17A) is a proinflammatory cytokine. It is known that IL-17 plays a central role in the activation of neutrophilic and macrophage in the lung in patients with COPD and severe BA [3, 7, 8]. IL-18 is one of the 11 members of the IL-1*β* family, and like IL-1*β*, it is mainly secreted by monocytes and macrophages, having the capability to quickly respond to external factors and trigger major proinflammatory reactions [3]. Overexpression of IL-18 in the airways in patients with COPD has been shown and can lead to emphysema, the development of fibrosis in the bronchi and blood vessels of the lungs, and the formation of pulmonary hypertension [7, 8]. Due to its T-helper type 2 cell- (Th-2-) inducing functions, IL-18 can also participate in inflammation and hyperreactivity of the respiratory tract in asthma and promote the recruitment of eosinophils to the airways [9–12]. On the other hand, IL-18 would further induce immune cells to produce a large amount of inflammatory factors to aggravate the disease [13, 14]. Thus, putting emphasis on the study of IL-18 in COPD is quite important.

As reported, oral NAC is a classical medicine to treat elderly COPD patients; it had multiple effects such as dissolving mucus, antioxidation, and anti-inflammation. However, whether NAC would have effect on IL-18 has not been fully clarified yet. So, in this study, we explored the treatment effect of NAC on COPD patients to see whether it would suppress IL-18 and further investigated the mechanism behind.

## 2. Method and Materials

### 2.1. Patients Enrolled in the Research

A total of 112 COPD patients and 103 health individuals were recruited in Jinshan Hospital, Fudan University, from May 2019 to March 2020. All COPD patients enrolled were treated with oral administration of NAC (acetylcysteine tablets, HaiNan ZangBang Pharmaceutical Co., Ltd., China) (1200 mg/day), and the medication lasted 100 days approximately (89-112 days). All participants signed the written informed consent. The study was conducted in accordance with the relevant guidelines and regulations developed by the aforementioned ethics committees. Our research was approved by the research ethics committees of Jinshan Hospital Affiliated to Fudan University, China (approval number: Jinshan Medical Ethics Research 2019-13-02).

The diagnosis of COPD was based on chronic obstructive pulmonary disease: diagnosis and management, and COPD grading was performed in accordance with the GOLD criteria [15, 16]. The inclusion criteria were showed as follows: (1) patients who were confirmed as COPD and in stable period; (2) patients received no antibiotics, glucocorticoids, oxygen therapy, and theophylline medications treatment within 2 weeks before enrolled in the research; and (3) patients who signed informed consent forms for voluntary participation in the research. The exclusion criteria were as follows: (1) patients with acute exacerbations which may affect the natural process of cytokine; (2) patients accompanied by pulmonary interstitial fibrosis, tuberculosis, bronchial pneumonia, and lung cancer; and (3) patients with major diseases of the nonrespiratory system, such as severe cardiovascular, cerebrovascular diseases and neurological diseases or liver and kidney dysfunction, and various tumors.

### 2.2. The Measurement of Cytokine by Enzyme-Linked Immunosorbent Assay (ELISA)

Patients' blood samples were centrifuged immediately after collection in order to separate serum, and approximately 1.5-2 ml of serum was collected from each patient. After separation, serum samples were immediately stored at −80°C. The cytokine concentration level was determined by using enzyme-linked immunosorbent assay (ELISA) kit (Sino Biological, China). The test was performed according to the manufacturer's instructions.

Mouse blood was immediately drawn after the mice were intraperitoneally anaesthetized with thiopental (70 mg/kg) and euthanized by transecting the abdominal aorta, centrifuged to obtain the serum. The mouse cytokine was measured by ELISA kit (Sino Biological, China). The test was performed according to the manufacturer's protocol as well.

### 2.3. Animals

C57BL/6 male mice (6–8 week old) were used in this study. The mice were divided into five groups, and every group contains 10 mice: Group 1—control group; Group 2—the animal model-cigarette smoke (CS) (Hongta Tobacco company, China) (20 cigarettes per day, for 60 min per session, six times per week)+lipopolysaccharide (LPS) (Abcam, Britain) (5 *μ*g/per mouse, 1time/week, from 3rd week to 8th week) group; Group 3—the animal model-CS+LPS+NAC (Abcam, Britain) (40 mM in the drinking water, NAC was administered from the 3th week till the end of the experiment) group; Group 4—the animal model-CS+LPS+anti-IL-18 group; and Group 5—the animal model-CS+LPS+IgG2A group. The animal experiment lasted for 8 weeks. All groups of mice were fed a standard diet and had free access to water. The protocol of animal experimental procedures was approved by the Ethics in Research Committee for Human and Animal Studies of Fudan University, School of Medicine.

### 2.4. Flow Cytometry Analysis

Bronchoalveolar lavage fluid (BALF) was obtained through the tracheal cannula by washing the mouse airway lumen with PBS. Then, the BALF was immediately centrifuged at 1500RPM for 5 min to get cell pellet. The cell type was further measured and determined by flow cytometry. The data analysis was performed on FlowJo (BD Bioscience, USA). The immunofluorescent antibodies used in the research were shown as follows: CD45-V500, CD11b-PerCP, F4/80-PE, CD206-BV421, CD3-FITC, and NK1.1-APC (BD Bioscience, USA). The following is the mouse macrophage: CD45^+^CD11b^+^F4/80^+^CD206^+^. Natural killer cells (NK) are as follows: CD45^+^CD3^−^NK1.1^+^. The related isotype antibodies were used as negative control. The result was analyzed with FlowJo 10.6.2 (BD Bioscience, USA).

### 2.5. Immunodepletion of IL-18

The anti-mouse IL-18 antibody was injected to delete the inner IL-18 in mice (50 *μ*g/mouse, R&D Systems, USA). Control mice were injected with a nonspecific antibody (IgG2A, R&D Systems, USA).

### 2.6. Western Blot

The experiment was conducted as previously described [17]. Cell lysate mixtures were resuspended in 40 *μ*l Laemmli Loading Buffer containing beta-mercaptoethanol (Bio-Rad Laboratories, CA) before Western blot analysis. Proteins were separated by sodium dodecyl sulfate polyacrylamide gel electrophoresis (SDS-PAGE) at 80 V before transferring to polyvinylidene fluoride (PVDF) membranes (Whatman Protran, 0.45 *μ*M) at 80 V (1.5 hours at 4°C). Membranes were blocked for 1 hour at room temperature using 1xTBST with 0.5% nonfat milk. Membranes were incubated for 16 hours at 4°C with the primary antibodies (1 : 1000), followed by a 1-hour incubation with a 1 : 10000 diluted secondary antibody. Blots were developed using enhanced chemiluminescence (ECL) kit (Invitrogen).

### 2.7. Histopathological Analysis

The upper left lungs of mice from each group were perfused and fixed with 5% formalin for 24 hours, and four-micrometer-thick slices were stained with hematoxylin and eosin for analysis. The result was evaluated by two investigators blindly, based on the histopathology score system, as previously descripted [18].

### 2.8. Statistical Analysis

Data was analyzed by SPSS software (20.0 IBM, USA). The significance of the results was tested by two-way ANOVA using GraphPad Prism 7.0 (GraphPad Software, San Diego, CA). All representative data were shown as the mean ± standard deviation (SD) from three separate experiments in triplicate. Comparisons between groups were analyzed by independent samples *t*-test. *P* < 0.05 was considered statistically significant.

## 3. Result

### 3.1. The Clinical Characteristic of Patients and Health Individuals Enrolled

A total of 112 COPD patients and 103 health individuals enrolled in the study. There was no clinical characteristic difference between these two groups. The basic information is shown in Table 1.

### 3.2. The Cytokine Expression in COPD Patients Changed Dramatically Compared with That in Health Individuals

We measured the inflammation-related cytokine in serum from both COPD patients and health individuals, including TGF-*β*, IL-1*β*, IFN-*γ*, IL-6, IL-10, TNF-*α*, and IL-18. The results showed that the contents of IL-1*β*, TNF-*α*, IFN-*γ*, IL-6, TGF-*β*, and IL-18 in serum had increased in COPD patients compared with health individuals, while IL-10 was decreased (Figure 1(a)). After NAC treatment, the levels of IL-1*β*, IFN-*γ*, TNF-*α*, and IL-18 in COPD patients' serum were decreased, and IL-10 was increased conversely; no obvious change of TGF-*β* and IL-6 was observed (Figure 1(b)). Further investigation demonstrated that before COPD patients had received medical treatment, the IL-18 had positive correlation with IFN-*γ* (*P* = 0.001), IL-1 (*P* = 0.024), and TNF-*α* (*P* = 0.020) and negative correlation with IL-10 (*P* = 0.003); besides, it had no correlation with other cytokines (Figure 1(c)); the result indicated that IL-18 had great connection with IFN-*γ*.

### 3.3. NAC Reduced IFN-*γ* and IL-18 in a COPD Mouse Model Induced by CS and LPS

We use C57BL/6 mice to establish a COPD mouse model. Cigarette smoking exposure and LPS were used to develop the COPD mouse model. In order to verify the expression of a variety of cytokines in COPD patients. The cytokines in serum were measured after the mice were killed. The result showed that the contents of IFN-*γ* and IL-18 increased in COPD mice compared with the control group, which was consistent with the result of COPD patients. On the other hand, IL-18 was found to be positively correlated with IFN-*γ* (Figure 2(a)). After the treatment of NAC, IL-18 and IFN-*γ* decreased significantly (Figure 2(b)).

In order to further explode the connection between IL-18 and IFN-*γ*, anti-IL-18 was used to delete the inner IL-18 in COPD mice (the elimination efficiency was measured by ELISA). The result showed that after eliminating IL-18 in COPD mice, IFN-*γ* also decreased greatly (Figure 2(c)). The experimental results above might give the hypothesis that NAC could reduce the expression of IFN-*γ* through depressing the level of IL-18 in mouse lungs.

### 3.4. NAC and Anti-IL-18 Alleviated the Inflammation and Injury in Mouse Lung Tissues Treated with CS and LPS

The model was next evaluated as well as the healing effect of NAC and anti-IL-18 to the inflammation in response to the treatment of CS combined with LPS in a mouse lung. As shown in Figure 3, the histological section was analyzed that compared with the control group, the CS and LPS treatment group presented more lung injury and inflammation; the number of immune cells infiltrating in lung tissues and airway was also larger. However, when the mice were cotreated with NAC, the inflammation was dramatically decreased, and the same phenomenon was also observed in the group of mice injected with anti-IL-18 as well, while the mice injected with IgG2 had no obvious change. The histopathological changes were evaluated by two investigators blindly based on a histopathology score system [18]. The result confirmed that NAC and anti-IL-18 could alleviate the inflammation and injury in a mouse lung induced by CS and LPS.

### 3.5. The Expression of IL-18 in Macrophages from BALF of COPD Mice Was Increased

Flow cytometry was used to evaluate the expression of IL-18 in macrophages in mouse lungs. The BALF from mice was obtained, and cells were collected and analyzed by flow cytometry immediately. As depicted in Figure 4, IL-18 was obviously higher in COPD mouse macrophages than in the normal control group. After NAC treatment, the IL-18 in macrophages was significantly decreased. Meanwhile, the IFN-*γ* in nature killer cells (NK) was decreased as well. In the anti-IL-18 group, the same phenomenon was also observed, which might indicate that the activation of NK cells and the release of IFN-*γ* were induced by IL-18 released from macrophages, and NAC could suppress IL-18 to alleviate the inflammation in lung and rebalance the immune status of mice.

### 3.6. NAC Suppressed IL-18 Expression in Mouse Macrophages through Downregulating NLRP3

Flow cytometry was then used to sort macrophages form BALF. The protein levels of human reactive inflammasome (NLRP3, AIM2, and NLRC4), cleaved caspase 1, and IL-18 in macrophages were further evaluated by Western blot (Figure 5). With LPS combined with CS treatment, NLRP3, cleaved caspase 1, and IL-18 in macrophages increased dramatically. However, after NAC treatment, the level of NLRP3, cleaved caspase 1, and IL-18 had significantly decreased, suggesting that NAC could effectively improve the immune status by down-regulating NLRP3 in macrophages to inhibit the synthesis of IL-18, which was a vital activator of IFN-*γ*.

## 4. Discussion

COPD was one of chronic respiratory diseases, and it becomes a major public health problem in the 21^st^ century, because of its high prevalence, morbidity, and mortality [19]. Nowadays, several pathology theories and relevant therapies about COPD were deeply investigated, among which inflammation and related cytokine were emphasized in clinical treatment [20]. Many immune cells and its mediators were involved in the inflammatory process of the disease, among which macrophages played a crucial role in the pathogenesis of COPD inflammation. Previous reports showed that IL-18 was a master regulator driving destructive and remodeling processes in the lungs of patients with COPD [21, 22]. So, in this study, we measured the level of IL-18 and other inflammation cytokines in COPD patients and the mouse COPD model. The truth was unveiled that in COPD patients, the inflammation was persisting in the lung as well as in the mouse model. Meanwhile, we found IL-18 had a great connection with other inflammation cytokines, especially IFN-*γ*, which indicated that IL-18 was an important factor in driving IFN-*γ* response and release. Thus, in order to further investigate the relationship between IL-18 and IFN-*γ* in the lung tissue, we established a mouse model of COPD, using an antibody to eliminate IL-18 in mice. After injection, the inflammation and lung injury in mouse lungs were relieved and the expression level of IFN-*γ* was significantly dropped. On the other hand, the expression of IFN-*γ* in NK cells decreased as well. Several researches revealed that IL-18 was a unique factor involved in the activation of various immune cells, including T cells and NK cells, via the simultaneous activation of the NF-*κ*B pathway [12, 23, 24]. Other researches reported that when IL-18 bound its receptors to form IL-18/IL-18R*α*/IL-18R*β* complex, it could induce phosphorylation of STAT3 in NK cells and the p38 MAP kinase pathway in neutrophils as well [25–27]. Our research demonstrated that IL-18 played a great role in inflammation procession indeed, and inflammation in the lung could be suppressed by reducing the expression level of IL-18, which might be an effective way to improve the inflammation status of COPD patients.

IL-18 has a fairly wide range of biological effects and exhibits pleiotropic properties in the immune response. High expression of IL-18 in the respiratory tract has been shown in patients with COPD and BA [3, 6–8, 25]. IL-18 serves as a cofactor for the development of both T-helper type 1 (Th1) and Th2 cells and can also increase NK activity and Fas-ligand expression in cells [25, 26]. It is shown that this cytokine exhibits the qualities of a strong conductor, enhancing the activation of various proinflammatory cytokines, including IFN-g, IFN-*γ*, GM-CSF, TNF-*α*, IL-13, IL8, IL-17, and IL-5 [23, 24]. Given the multifaceted proinflammatory nature of IL-18 activity, the detected elevated serum concentrations of this cytokine suggest that IL-18 plays an important role in the implementation of systemic inflammation in both COPD and BA and also in the asthma-COPD overlap (ACO). The revealed correlations between serum levels of IL-17, IL-18, and TNF-*α* and lung function parameters in the examined patients may signify the effect of these cytokines on the development of pathophysiological mechanisms in these obstructive diseases [6, 23–27]. NAC is a kind of sulphur-containing amino acid and antioxidant and could be used as a classical drug for the treatment of COPD and other variety of diseases, which is easily available in many countries. It provides the sulfhydryl groups and acts both as a precursor of reduced glutathione and as a direct reactive oxygen species (ROS) scavenger, hence modulating the redox status in the cells, thus influencing many inflammation pathways [28]. Pervious reported showed that NAC could directly influence several signaling pathways such as NF-*κ*B, p38, ERK1/2, SAPK/JNK, c-Jun, and c-Fos to adjust immune status [29–32]. However, whether NAC could affect macrophages and IL-18 had not been fully clarified. As a member of the IL-1 family, the IL-18 precursor is processed intracellularly by caspase 1 into its biologically mature molecule of 18 kDa [33]. It is known that chronic inflammation has been shown as a key player at different stages of COPD, and a prominent signaling pathway for acute and chronic inflammation is the activation of the caspase 1 inflammasomes, which are reported as a group of cytosolic protein complexes formed to mediate host immune responses to microbial infection and cellular damage, among which NLRP3, AIM2, and NLRC4 are of great importance in the context of COPD for their activities in modulating immune responses [34–36]. In our research, after taking NAC, the IL-18 in both serum and macrophages in COPD mice was dramatically decreased, a histological section showed inflammation, and lung injury subsided effectively. Meanwhile, the protein of inflammasomes and cleaved caspase 1 in macrophages was measured by Western blot before and after the COPD mice taking NAC. The result suggested the NAC could downregulate the expression of NLRP3 in macrophages, thus reducing the synthesis of IL-18. In summary, somehow, NAC might intervene the ability of macrophages to produce IL-18 by downregulating the expression of inflammasomes to improve the inflammation in the lung of COPD patients.

In conclusion, our paper was the first to find the effect of NAC on macrophages in suppressing the release of IL-18. The hypothesis was further demonstrated based on the mouse COPD model. NAC could influence the inflammasomes in macrophages to downregulate the synthesis of IL-18, thus improving the immune and inflammation status (Figure 6). Of course, further investigation will be required to fully describe the specific mechanisms of NAC on macrophages in regulating inflammasome-related protein.

## Figures and Tables

**Figure 1:** The expression of variety of cytokines in COPD and health individuals. (a) The contents of TGF-*β*, IL-1*β*, IFN-*γ*, IL-6, IL-10, TNF-*α*, and IL-18 in the serum from COPD patients and health individual. (b) After NAC treatment, the expression level of TGF-*β*, IL-1*β*, IFN-*γ*, IL-6, IL-10, TNF-*α*, and IL-18 in serum of COPD patients. (c) The correlation between IL-18 and other cytokines in COPD patients before taking NAC. Note: ^∗^*p* ≤ 0.05, ^∗∗^*p* ≤ 0.01, and ^∗∗^*p* ≤ 0.001.

**Figure 2:** The expression level of IL-18 and IFN-*γ* in a COPD mouse model. (a) The contents of IFN-*γ* and IL-18 in the serum from COPD mouse and the correlation between these two cytokines. (b) The expression level of IL-18 and IFN-*γ* in the serum from COPD mouse before and after taking NAC. (c) The expression level of IFN-*γ* and IL-18 in the serum from COPD mouse after injection with anti-IL-18 and Ig-G2 control. Note: ^∗^*p* ≤ 0.05, ^∗∗^*p* ≤ 0.01, and ^∗∗^*p* ≤ 0.001.

**Figure 3:** NAC and IL-18 alleviated the inflammation and the injury induced by CS and LPS in mouse lung. (a) H&E staining of lung tissue from every group. Scale bar: 20 *μ*m. (b) Lung injury scores were evaluated. Note: ^∗^*p* ≤ 0.05, ^∗∗^*p* ≤ 0.01, and ^∗∗^*p* ≤ 0.001.

**Figure 4:** IL-18 in macrophages and IFN-*γ* in NK cells were measured by flow cytometry in different group of mice, including COPD mice, mouse with NAC treatment, and mouse with injection with IL-18 and IgG2. Note: ^∗^*p* ≤ 0.05, ^∗∗^*p* ≤ 0.01, and ^∗∗^*p* ≤ 0.001.

**Figure 5:** The protein expression of inflammasome-related markers, cleaved caspase 1, and IL-18 was measured by Western blot in macrophages in different groups of mice.

**Figure 6:** Simple diagram explaining the mechanism of NAC working on macrophages.

**Table 1:** The clinical information of individuals enrolled in the study.

	COPD	Health control	*p*
Age			
≤60	33	38	0.310
>60	79	65	
Gender			
Male	66	65	0.674
Female	46	38	
BMI (kg/m^2^)	26.21 ± 4.33	25.55 ± 5.02	0.467
Smoking status			
Yes	72	73	0.312
No	40	30	
Smoking index			
0-200	76	68	0.580
>200	36	35	
Score of mMRC	2.66 ± 0.92		
Clinical history of COPD			
≤10	33		
>10 ≤ 20	45		
>20	34		

## Data Availability

All the data can be accessed by e-mailing the corresponding author for request.
